The article "Maintenance of Stemness in Oxaliplatin-Resistant Hepatocellular Carcinoma Is Associated with Increased Autocrine of IGF1" was retracted in 2025. Reasons: errors in the data; errors in the images; duplicated images; overlap with earlier publications.

# Maintenance of Stemness in Oxaliplatin-Resistant Hepatocellular Carcinoma Is Associated with Increased Autocrine of IGF1

**DOI:** 10.1371/journal.pone.0089686

**Published:** 2014-03-14

**Authors:** Yang Bu, Qing-An Jia, Zheng-Gang Ren, Ju-Bo Zhang, Xue-Mei Jiang, Lei Liang, Tong-Chun Xue, Quan-Bao Zhang, Yan-Hong Wang, Lan Zhang, Xiao-Ying Xie, Zhao-You Tang

**Affiliations:** 1 Institutes of Biomedical Sciences, Fudan University, Shanghai, China; 2 Liver Cancer Institute, Zhongshan Hospital, Fudan University, Key Laboratory of Carcinogenesis and Cancer Invasion, Ministry of Education, Shanghai, China; 3 Hepatobiliary Surgery, Shanxi Provincial People's Hospital, Xi'an, China; 4 Department of Gastroenterology, Haikou People's Hospital, Haikou, China; University of Hong Kong, Hong Kong

## Abstract

**Background:**

Evidence suggests that many types of cancers are composed of different cell types, including cancer stem cells (CSCs). We have previously shown that the chemotherapeutic agent oxaliplatin induced epithelial-mesenchymal transition, which is thought to be an important mechanism for generating CSCs. In the present study, we investigate whether oxaliplatin-treated cancer tissues possess characteristics of CSCs, and explore oxaliplatin resistance in these tissues.

**Methods:**

Hepatocellular carcinoma cells (MHCC97H cells) were subcutaneously injected into mice to form tumors, and the mice were intravenously treated with either oxaliplatin or glucose. Five weeks later, the tumors were orthotopically xenografted into livers of other mice, and these mice were treated with either oxaliplatin or glucose. Metastatic potential, sensitivity to oxaliplatin, and expression of CSC-related markers in the xenografted tumor tissues were evaluated. DNA microarrays were used to measure changes in gene expression as a result of oxaliplatin treatment. Additionally, an oxaliplatin-resistant cell line (MHCC97H-OXA) was established to assess insulin-like growth factor 1 secretion, cell invasion, cell colony formation, oxaliplatin sensitivity, and expression of CSC-related markers. The effects of an insulin-like growth factor 1 receptor inhibitor were also assessed.

**Results:**

Oxaliplatin treatment inhibited subcutaneous tumor growth. Tumors from oxaliplatin-treated mice that were subsequently xenografted into livers of other mice exhibited that decreasing sensitivity to oxaliplatin and increasing pulmonary metastatic potential. Among the expression of CSC-related proteins, the gene for insulin-like growth factor 1, was up-regulated expecially in these tumor tissues. Additionally, MHCC97H-OXA cells demonstrated that increasing cell invasion, colony formation, and expression of insulin-like growth factor 1 and CSC-related markers, whereas treatment with an inhibitor of the insulin-like growth factor 1 receptor suppressed these effects.

The article "Maintenance of Stemness in Oxaliplatin-Resistant Hepatocellular Carcinoma Is Associated with Increased Autocrine of IGF1" was retracted in 2025. Reasons: errors in the data; errors in the images; duplicated images; overlap with earlier publications.

**Conclusion:**

Maintenance of stemness in oxaliplatin-resistant hepatocellular carcinoma cells is associated with increased autocrine of IGF1.

## Introduction

Liver cancer, most commonly hepatocellular carcinoma (HCC), is the fifth most frequently diagnosed cancer in men worldwide, but the second-most frequent cause of cancer death. It is also the 7th-most diagnosed and the 6th-most cause of cancer death in women, according to Jemal et al [1]. In clinical practice, fewer than 30% of patients with HCC can be treated with curative options such as liver transplantation, surgical resection, and ablation therapy, because it is at an advanced stage when the cancer have been diagnosed [2]. As a result, transcatheter hepatic arterial chemoembolization (TACE) and systemic chemotherapy are frequently used [3], [4]. HCC, however, is well known to be relatively chemotherapy-resistant. In a phase II study of the use of the chemotherapeutic agent oxaliplatin to treat unresectable, metastatic, or recurrent HCC, only 47% of patients exhibited disease stabilization of short duration [5]. Furthermore, side effects of tumor chemotherapy often reports, which is a major obstacle to restricting the long-term effect of chemotherapy[6], [7], [8], [9], [10], [11]. Cancer recurrence is frequently seen in patients who have undergone chemotherapy, and these recurrent cancers have been shown to be both highly malignant and drug-resistant. Recent evidence suggests that many cancers, including HCC, are hierarchically organized into a variety of different cell types, including a subset of stem cell-like cells capable of self-renewal and thought to be responsible for most recurrences and metastases [12], [13], [14], [15]. These cancer stem cells (CSCs) are resistant to conventional chemotherapy due to characteristics such as high expression of drug transporters, relative cell cycle quiescence, high levels of DNA repair, and resistance to apoptosis [16], [17]. Costello et al [18] found that human acute myeloid leukemia CD34+/CD38− progenitor cells exhibited that decreasing sensitivity to daunorubicin (a chemotherapeutic agent) compared with CD34+/CD38+ cells, as well as high expression levels of the drug resistance-related genes LRP and MRP. Similarly, Liu et al [19] reported that CD133+ glioblastoma cells treated with multiple chemotherapeutic agents had fewer deaths than their CD133− counterparts as a result of overexpression of anti-apoptotic genes such as FLIP, Bcl-2, and Bcl-XL. The existence of CSCs that possess the ability to seed new tumors may explain why chemotherapy for tumor often initially appears successful, but ultimately fails to prevent cancer recurrence.

The article "Maintenance of Stemness in Oxaliplatin-Resistant Hepatocellular Carcinoma Is Associated with Increased Autocrine of IGF1" was retracted in 2025. Reasons: errors in the data; errors in the images; duplicated images; overlap with earlier publications.

Insulin-like growth factor 1 (IGF1) mediates various cellular processes, and the activation of insulin-like growth factor 1 receptor (IGF1R) has been associated with increased tumorigenesis, metastasis, and resistance to existing forms of cancer treatment [20], [21], [22], [23]. The binding of IGF1 to IGF1R leads to the activation of multiple cell survival signaling pathways [24], [25]. Lee J et al [26] reported that IGF-1 treatment increased the levels of β-catenin and cyclin D1 but decreased the levels of E-cadherin, which is one of the most important characteristics of epithelial-mesenchymal transition (EMT). Protein kinase B negatively regulates glycogen synthase kinase-3b, thus promoting β-catenin-induced stem cell self-renewal [27]. The mitogen-activated protein kinases/extracellular signal-regulated kinases (MAPK/ERK) signaling pathway has also been shown to play a role in CSC self-renewal and tumorigenicity in a number of cancers [28], [29].

The objective of this study was to explore how oxaliplatin-resistant HCC retains oxaliplatin resistance even after a series of passages without oxaliplatin treatment. DNA microarrays were used to evaluate gene expression in cancer tissue from oxaliplatin-treated and control mice. We found that the gene encoding IGF1 was significantly up-regulated in tumors from oxaliplatin-treated mice. We also demonstrated that stem cell-like characteristics of the cancer cells are regulated by IGF1 in an autocrine manner.

## Materials and Methods

### Reagents and antibodies

Oxaliplatin and the IGF1R inhibitor PQ401 were purchased from Sigma Chemical Company (St Louis, MO, USA). For antibodies used in immunoblotting and/or immunochemistry were purchased as follows: mouse anti-human monoclonal cluster of differentiation (CD)44 (Abcam, Cambridge, MA, USA), used at concentration of 5 μg/ml; rabbit anti-human monoclonal CD90 (Abcam), used at concentration of 1 μg/ml; mouse anti-human monoclonal epithelial cell adhesion molecule (EpCAM) (Abcam), used at concentration of 5 μg/ml; mouse anti-human monoclonal aldehyde dehydrogenase (ALDH) (Abgent, San Diego, CA, USA), used at concentration of 3 μg/ml; mouse anti-human monoclonal β-catenin (Abcam), used at concentration of 2 μg/ml; mouse anti-human monoclonal IGF1 (Abcam), used at concentration of 1 μg/ml; rabbit anti-human monoclonal (sex determining region Y)-box 2 [Homo sapiens (human)] (SOX2) (Abcam), used at 1∶500 dilution; mouse anti-human monoclonal octamer-binding transcription factor 4 (OCT4) (Abcam), used at 1∶100 dilution; mouse anti-human monoclonal E-cadherin (Abcam), used at 1∶100 dilution; mouse anti-human monoclonal vimentin (Abcam), used at concentration of 3 μg/ml; and rabbit anti-human monoclonal β-actin (Epitomics, Burlingame, CA, USA), used at 1∶1000 dilution.

The article "Maintenance of Stemness in Oxaliplatin-Resistant Hepatocellular Carcinoma Is Associated with Increased Autocrine of IGF1" was retracted in 2025. Reasons: errors in the data; errors in the images; duplicated images; overlap with earlier publications.

### Animal treatment

BALB/c nu/nu mice (aged 4–6 weeks and weighing approximately 20 g) were obtained from the Chinese Academy of Sciences and maintained under standard pathogen-free conditions. All mice were handled in accordance with the recommendations of the National Institutes of Health Guidelines for Care and Use of Laboratory Animals. Before all the operations, the mice were subjected to intraperitoneal anesthesia and killed by dislocating spine finally. The experimental protocol used was approved by the Shanghai Medical Experimental Animal Care Commission. The high-metastatic-potential human HCC cells used in this study were MHCC97H cells, which were established in our institution [30]. MHCC97H cells (5×10^6^ cells per mouse) were injected subcutaneously (s.c.) into the upper left flank region of each of 12 mice to produce tumors. Seven days later, half of the mice were treated with 0.1 ml oxaliplatin (10 mg/kg) via tail vein injection once a week, and the other half were similarly injected with 0.1 ml 5% glucose solution (GS) as a control. Four weeks later, orthotopic xenografts were measured and performed as described in previous publication [31], [32].The s.c. tumors were removed respectively, randomly selected tumor tissues of one mouse from each group and minced into equal size of 2 mm^3^, and randomly transplanted into the livers of additional 24 mice. Among these, 12 mice received tumor tissues from GS group, and the other 12 from oxali group. Half of the mice from each GS or oxali group were then treated with GS or oxaliplatin as above. As a result, four study groups were formed: GS/GS, oxali/GS; GS/oxali, oxali/oxali. Another five weeks later, residual HCC tissues were collected from the mice, the metastatic potential and oxaliplatin sensitivity of residual HCC tissue of the orthotopic xenografts were evaluated.

### Immunohistochemical analysis

The expression levels of stemness-related markers in tumors from oxaliplatin- and GS-treated s.c. tumor mice were determined by immunohistochemistry. Tumor tissues were fixed, embedded, and sliced into 5-μm thick sections. Immunohistochemical staining of the proteins CD44, ALDH, SOX2, OCT4, E-cadherin, EpCAM, vimentin, β-catenin, and IGF1 was performed using a standard protocol [33].

### DNA microarray analysis

DNA microarrays were used to evaluate changes in gene expression.Total RNA was extracted from HCC tissue from both oxaliplatin- and GS-treated s.c. tumor mice, and three independent isolations and microarray analyses were performed using 4×44K human Genome Array chips (Agilent Whole Human Genome Oligo Microarray Kit, Agilent Technologies, Santa Clara, CA, USA) according to the manufacturer's instructions. Data analysis was performed using feature extraction and GeneSpring 12.0 software (Agilent Technologies). All data had uploaded GEO, and GEO accession number is GSE51951.

The article "Maintenance of Stemness in Oxaliplatin-Resistant Hepatocellular Carcinoma Is Associated with Increased Autocrine of IGF1" was retracted in 2025. Reasons: errors in the data; errors in the images; duplicated images; overlap with earlier publications.

### Enzyme-linked immunosorbent assays (ELISAs) to assess IGF1 levels in MHCC97H and MHCC97H-OXA cells

Levels of IGF1 in the culture supernatants and in the cell lysates were quantified by ELISA kits (R&D Lab Inc., Minneapolis, MN, USA). Oxaliplatin-resistant MHCC97H cell line was constructed as follow: MHCC97H cells grown to 60–70% confluence, which were harvested with trypsin and plated in T25 cell culture flasks (5×10^5^ cells per flask). After 24 h, the medium was replaced with DMEM containing 10% FBS and 2 μmol/l oxaliplatin. After 48 h, the medium was changed and drug treatment was terminated. Cells were allowed to recover, and when the surviving populations reached 80% confluence, cells were passaged and exposed to 2 μmol/l oxaliplatin again for 48 h. As cells became resistant to oxaliplatin, the above procedure was repeated using 5 μmol/l concentration of oxaliplatin. Until 25 μmol/l oxaliplatin were used, the cells were becoming stable resistant to oxaliplatin and re-named MHCC97H-OXA cells. Quadruplicate assays were performed according to the manufacturer's instructions and as described previously [34]. Absorbance was measured at 450 nm using a microplate spectrophotometer (Multiskin spectrum, Thermo Cooperation, America).

### Effects of PQ401 on Growth of MHCC97H cells

The proliferation of MHCC97H cells were assessed with Cell Counting Kit-8 (CCK8; Dojindo Molecular Technologies Inc., Kumamoto, Japan). MHCC97H cells were plated in 96-well plates (5×10^3^ cells per well) in DMEM supplemented with 10% FBS overnight, and were then treated with various concentrations of PQ401(10 mg PQ401 was dissolved with 1 ml DMSO and one tenth of the mixture was diluted 100-fold in DMEM, which is used as PQ401 stock solution) for 0,1, 2, 3 day. Then, the CCK8 reagent was added to each well according to the manufacturer's instructions. Results were expressed as the absorbance of each well at 450 nm as measured using a microplate spectrophotometer (Multiskin spectrum, Thermo Cooperation, America).

### Effects of Oxaliplate and PQ401 on MHCC97H-OXA and MHCC97H

To investigate the sensitivities of MHCC97H and MHCC97H-OXA cells to oxaliplatin, Cell Counting Kit-8 (CCK8; Dojindo Molecular Technologies Inc., Kumamoto, Japan) was used. Cells were plated in 96-well plates (3×10^3^ cells per well) and exposed to oxaliplatin at increasing concentrations (0, 2, 4, 8, 16, 32, 64, 128, 256 μmol/l) for 24, 48, 72, and 96 h. The CCK8 reagent was added to each well according to the manufacturer's instructions. Results were expressed as the absorbance of each well at 450 nm as measured using a microplate spectrophotometer (Multiskin spectrum, Thermo Cooperation, America). Meanwhile, to investigating the effects of IGF1R inhibitor PQ401, the same two groups of cells were digested and plated in T25 cell culture flasks (5×10^5^ cells per flask). After 24 h, the medium was replaced with DMEM containing 10%FBS and 10 μmol/l PQ401, the cells were cultured for 24 h continually. Then, repeating the above steps. According to mean of three experiments, calculating 50% cells growth inhibition (IC_50_) of every group.

The article "Maintenance of Stemness in Oxaliplatin-Resistant Hepatocellular Carcinoma Is Associated with Increased Autocrine of IGF1" was retracted in 2025. Reasons: errors in the data; errors in the images; duplicated images; overlap with earlier publications.

### Cell invasion assays

Invasion of MHCC97H and MHCC97H-OXA cells was assessed by transwell assays using Boyden chambers (Corning, Tewksbury, MA, USA). Briefly, 80 μl matrigel (BD Biosciences, San Jose, CA, USA) was added to each well 6 h before cells were seeded on the membrane. Cells (6×10^4^ cells, per well) in serum-free DMEM were seeded into the upper chamber of each well of 24-well plates containing 8.0-μm pore size membranes. DMEM containing 10% FBS was added to the lower chamber of each well. After 48 h, cells that had reached the underside of the membrane were stained with Giemsa (Sigma Chemical Company), counted, and photographed at ×200 magnification. To investigate the effect of IGF1R inhibitor PQ401, the invasion assay was repeated except that DMEM containing 10% FBS and 10 μmol/l PQ401 was added to the lower chamber of each well of MHCC97H-OXA cells.

### Cell colony formation assays

MHCC97H or MHCC97H-OXA cells (1×10^3^ cells per well) were plated in 6-well plates (Corning) and cultured with DMEM containing 1% FBS. Culture medium was replaced every 3 d, and the colonies were fixed with ice-cold 4% paraformaldehyde after 14 days. Cells were stained with Giemsa (Sigma Chemical Company) and photographed at ×5 magnification. To investigate the effect of IGF1R inhibitor PQ401, the assay was repeated except that MHCC97H-OXA cells were exposed to DMEM containing 1% FBS and 10 μmol/l PQ401.

### Immunofluorescence assays

Expression of E-cadherin, vimentin, CD44, and CD90 in MHCC97H and MHCC97H-OXA cells was determined by immunofluorescence as previously described [33]. Cells were grown to 20–30% confluency on glass cover slips in DMEM supplemented with 1% FBS and then fixed, permeabilized, blocked, and incubated with the appropriate antibodies overnight at 4°C. Slides were then washed and incubated with CY3-conjugated secondary antibody (Jackson Labs, Bar Harbor, ME, USA). Cells were counterstained with 4′-6-diamidino-2-phenylindole to visualize cell nuclei and imaged using fluorescence microscopy (Olympus, Tokyo, Japan). To investigate the effect of IGF1R inhibitor PQ401, MHCC97H-OXA cells were cultured similarly except that DMEM containing 1% FBS and 10 μmol/l PQ401 was used.

The article "Maintenance of Stemness in Oxaliplatin-Resistant Hepatocellular Carcinoma Is Associated with Increased Autocrine of IGF1" was retracted in 2025. Reasons: errors in the data; errors in the images; duplicated images; overlap with earlier publications.

### Western blots

Western blots were performed to assess the expression of CD44, CD90, SOX2, OCT4, E-cadherin, vimentin, and β-actin in MHCC97H, MHCC97H-OXA, and 10 μmol/l PQ401-treated MHCC97H-OXA cells. The protein extracts of the cells were determined using the BCA Protein Assay Kit (Beyotime Institute of Biotechnology, Shanghai, China) according to the manufacturer's instructions [33].

### Statistical analysis

Quantitative differences in the data on tumor volume, pulmonary metastasis nodules, gene and protein expression levels, cell invasiveness, colony formation, and oxaliplatin sensitivity were evaluated by t-test. Statistical analysis was performed using SPSS 15.0 software for Windows (SPSS Inc. Chicago, IL, USA). P<0.05 was considered statistically significant.

## Results

### Oxaliplatin treatment inhibited s.c. tumor growth, but failed to inhibit growth of xenografted liver tumors; increased pulmonary metastasis was seen in xenografted liver tumors that originated as s.c. tumors from oxaliplatin-treated mice

Based on average tumor weights, intravenous oxaliplatin treatment significantly inhibited s.c. tumor growth (3.20±0.14 g for GS group vs. 1.58±0.29 g for oxali group, P = 0.0005) (Figure 1A). When s.c. tumors from GS group were orthotopically xenografted into the livers of other 12 mice, oxaliplatin treatment also inhibited liver tumor growth (2.81±0.25 g for GS/GS group vs. 1.89±0.42 g for oxali/GS group, P = 0.0011) (Figure 1B). Additionally, s.c. tumors from oxali group mice that were orthotopically xenografted into the livers of another 12 mice, the recipient mice showed resistance to oxaliplatin treatment (1.82±0.21 g for GS/oxali group vs. 1.68±0.27 g for oxali/oxali group, P = 0.315) (Figure 1C). Furthermore, oxali/oxali group significantly (P = 0.0013) increased the number of pulmonary metastasis (51.24±19.87) compared with oxali/GS group (31.12±16.62) (Figure 1D).

**Figure 1:** Oxaliplatin treatment in vivo experiments. (A) Oxaliplatin treatment significantly inhibited the MHCC97H cells s.c. tumor. (B) GS-treated MHCC97H cells s.c. tumors were orthotopically transplanted into livers of other mice, and oxaliplatin treatment of these mice still produced significant therapeutic effects on the tumor tissues. (C) Oxaliplatin-treated MHCC97H cells s.c. tumors were orthotopically transplanted into livers of another mice, and oxaliplatin retreatment of these mice produced no significant therapeutic effects on the tumor tissues. (D) Oxaliplatin-treated MHCC97H cells s.c. tumors were orthotopically transplanted into livers of other mice, and these mice were retreated with oxaliplatin. These mice exhibited increasing pulmonary metastasis compared to the same treatment xenografts from GS-treated MHCC97H cells s.c. tumors (The top are fluorescence microscope photographs of lung tissues, below are Hematoxylin and eosin staining of lung metastasis sections, original magnification×100). Columns, mean of tumor weight of every group; Points, mean of lung metastasis numbers of two groups; bars, SD.

The article "Maintenance of Stemness in Oxaliplatin-Resistant Hepatocellular Carcinoma Is Associated with Increased Autocrine of IGF1" was retracted in 2025. Reasons: errors in the data; errors in the images; duplicated images; overlap with earlier publications.

### HCC tissue from oxaliplatin-treated s.c. tumor mice showed increased expression of stemness-related markers

Immunohistochemical staining (Figure 2) revealed that increasing proportions of CD44-, ALDH-, and EpCAM-positive CSCs in tumor tissue from oxaliplatin-treated s.c. tumor mice compared with GS-treated s.c. tumor mice. Significantly increased expression of SOX2 and OCT4, which are related to maintenance of stemness, was also observed after oxaliplatin treatment. The expression of vimentin and β-catenin, which are related to EMT, was also up-regulated in tumors from oxaliplatin-treated s.c. tumor mice. IGF1 expression was also significantly increased. In addition, the typical membranous E-cadherin expression was significantly down-regulated in tumors from oxaliplatin-treated s.c. tumor mice.

**Figure 2:** The s.c. tumor tissue by immunohistochemical. Tumor harvested from Oxaliplatin-treated s.c. tumor tissue and GS-treated s.c.tumor tissue (control) were fixed, embedded, sectioned, and applied to CSC- and EMT-related markers immunohistochemical staining, IgG were negative control groups, the nuclei or cytoplasm of positive cells were brownish, original magnification×200.

### Gene expression profiles in tumors from oxaliplatin-treated s.c. tumor mice were different from those of GS-treated s.c. tumor mice

The expression of 41,096 genes (Figure 3A) in liver tumor tissues from oxaliplatin- and GS-treated s.c. tumor mice was compared in three independent experiments. Gene expression in tumors from oxaliplatin- and GS-treated s.c. tumor mice had both similarities and differences. Expression profiles for 332 genes had >2-fold differences between oxaliplatin- and GS-treated s.c. tumor mice groups. Genes specifically up- and down-regulated in tumors from oxaliplatin-treated s.c. tumor mice included those related to chemokines, chemokine receptors, signal transduction, inflammation, proliferation, development, and metabolism. There were 267 up-regulated and 65 down-regulated genes. Some genes were closely related to the malignant phenotype of the tumor, such as IGF1, CXCR7, TCF3, NPR1, FGF18, DDR2, GLI2, CYR61, COL14A1, HSPH1, SOX11, TRIB2, PDZK1, and MMP2. IGF1 was selected as a target gene for further study. Both Immunohistochemical analysis (Figure 3B) and Western blot (Figure 3C) verified that the expression of IGF1 in tumors from oxaliplatin-treated s.c. tumor mice was significantly up-regulated.

The article "Maintenance of Stemness in Oxaliplatin-Resistant Hepatocellular Carcinoma Is Associated with Increased Autocrine of IGF1" was retracted in 2025. Reasons: errors in the data; errors in the images; duplicated images; overlap with earlier publications.

**Figure 3:** Gene expression profiles of tumor tissues from oxaliplatin-treated and GS-treated s.c. tumor (control). (A) 332 genes had more than 2-fold differences between oxaliplatin-treated and GS-treated s.c. tumor. (B) Immunohistochemical analysis revealed up-regulated expression of IGF1 in tumors from oxaliplatin-treated s.c. tumor, IgG were negative control groups, the cytoplasm of positive cells were brownish, original magnification×200. (C) Western blot analysis showed up-regulated expression of IGF1 in tumors from oxaliplatin-treated s.c. tumor.

### MHCC97H-OXA cells showed increasing secretion of IGF1

MHCC97H-OXA cells were morphologically distinguished from parental MHCC97H cells, demonstrating a spindle shape and increased formation of pseudopodia in place of the typical epithelial cell characteristics (Figure 4A). ELISAs revealed that the secretion of IGF1 in MHCC97H-OXA cells were increased significantly, which compared with parental MHCC97H cells (5307.44±301.75 pg/ml vs. 2905.44±362.93 pg/ml, P = 0.0000) (Figure 4B).

**Figure 4:** The difference between MHCC97H cells and MHCC97H-OXA cells. (A) MHCC97H-OXA cells were morphologically distinguished from parental MHCC97H cells, demonstrating a spindle shape and increasing formation of pseudopodia in place of epithelial cell characteristics. (B) ELISAs showed increased secretion of IGF1 in MHCC97H-OXA cells compared with parental MHCC97H cells. Columns, mean of three experiments; bars, SD.

### MHCC97H-OXA cells enhanced resistance to chemotherapy, which could be decreased by PQ401

The IGF1R inhibitor PQ401 inhibited the growth of MHCC97H, which positively correlated with drug concentration and duration. With our protocol, PQ401, at concentrations>15 μmol/l significantly reduced proliferation, at concentrations in the range of 10 μmol/l, had almost no effect on proliferation of MHCC97H cells (Figure 5A). The resistance of MHCC97H-OXA cells to oxaliplatin was increased over that of MHCC97H cells; the concentration of IC_50_ was higher in MHCC97H-OXA cells than in MHCC97H cells (84.67±8.50 μmol/l vs. 27.67±4.51 μmol/l, P = 0.0001). Meanwhile, treatment with PQ401 decreased the resistance of MHCC97H-OXA cells to oxaliplatin as demonstrated by reduction of IC_50_ (84.67±8.50 μmol/l vs. 18.37±3.96 μmol/l, P = 0.0000). There was no difference between MHCC97H cells and early incubation of MHCC97H cells with 10 μmol/l PQ401 in the resistance to oxaliplatin (Figure 5B).

The article "Maintenance of Stemness in Oxaliplatin-Resistant Hepatocellular Carcinoma Is Associated with Increased Autocrine of IGF1" was retracted in 2025. Reasons: errors in the data; errors in the images; duplicated images; overlap with earlier publications.

**Figure 5:** Effect of PQ401 on proliferation of parental MHCC97H and Oxaliplatin treatment of MHCC97H-OXA and parental MHCC97H cells. (A) MHCC97H cells were incubated with varying concentrations of PQ401, beginning on 0 day. Proliferative capacity was reflected by absorbance values (O.D.) on 0, 1, 2, 3 day. Columns, mean of three experiments; bars, SD; *, proliferation significantly reduced versus controls (containing 0.1% DMSO). (B) MHCC97H, MHCC97H-OXA cells in basal medium, another MHCC97H, MHCC97H-OXA cells in medium supplemented with 10 μmol/l PQ401, were cultured for 24 hours in advance. Then, the cells of four groups were incubated with varying concentrations of Oxaliplatin for 24 h, 48 h, 72 h, 96 h, and using CCK8 assay to calculate IC_50_ value of every group. Columns, mean of three experiments; bars, SD; **, P<0.001.

### MHCC97H-OXA cells showed enhancing invasion and cell colony formation, which could be attenuated by PQ401

The cell invasion assays (Figure 6A) demonstrated that MHCC97H-OXA cells passed through the basement membrane more efficiently than parental MHCC97H cells, based on the average number of cells crossing the basement membrane (44.33±8.67 *vs.* 22.17±7.44, *P* = 0.0009). The enhanced invasion of MHCC97H-OXA cells was inhibited by IGF1R inhibitor PQ401 treatment, as demonstrated by a decreased number of cells crossing the basement membrane (44.33±8.67 *vs.* 8.33±3.01, *P* = 0.0001). In colony formation assays (Figure 6B), MHCC97H-OXA cells exhibited a significantly higher colony-forming ability compared with parental MHCC97H cells, as measured by number of colony forming (53.83±8.70 *vs.* 27.17±8.30, *P* = 0.0003).Enhanced colony-forming ability of MHCC97H-OXA cells could be inhibited by PQ401, as demonstrated by a decreased number of colony forming (53.83±8.70 *vs.* 21.00±6.60, *P* = 0.0001).

**Figure 6:** MHCC97H-OXA cells enhanced invasion and cell colony formation, which was inhibited by treatment with IGF1R inhibitor PQ401. (A) The cell invasiveness assay demonstrated that the number of cells crossing the basement membrane was higher for MHCC97H-OXA cells than for MHCC97H cells, and was inhibited by PQ401 treatment, original magnification×200. (B) In colony formation assays, MHCC97H-OXA cells exhibited a significantly greater colony-forming ability compared with parental MHCC97H cells, likewise this was inhibited by PQ401 treatment, original magnification×5. (C) Column, mean of three experiments; bars, SD.

The article "Maintenance of Stemness in Oxaliplatin-Resistant Hepatocellular Carcinoma Is Associated with Increased Autocrine of IGF1" was retracted in 2025. Reasons: errors in the data; errors in the images; duplicated images; overlap with earlier publications.

### MHCC97H-OXA cells showed increasing expression of CSC-related markers, which could be suppressed by PQ401

To investigate the roles of oxaliplatin and PQ401 in modulating the expression of CSC-related markers, we examined the levels of expression in MHCC97H, MHCC97H-OXA, and PQ401-treated MHCC97H-OXA cells. In immunofluorescence assays (Figure 7A), we observed an increased expression of CSC-related markers CD44 and CD90 in MHCC97H-OXA cells; this change was inhibited by PQ401 treatment. In Western blots (Figure 7B), concentrations of the CSC- and EMT-related markers CD44, CD90, OCT4, SOX2, EpCAM, and vimentin were increased in MHCC97H-OXA cells, and decreased after treatment with PQ401. In addition, the typical membranous E-cadherin expression was significantly down-regulated in MHCC97H-OXA cells and up-regulated after treatment with PQ401.

**Figure 7:** MHCC97H-OXA cells increased expression of CSC-related markers, which was suppressed by treatment with the IGF1R inhibitor PQ401. (A) In the immunofluorescence assay, CSC- and EMT-related markers were up-regulated in MHCC97H-OXA cells, and these were attenuated by PQ401 treatment. (B) In Western blot analyses, CSC- and EMT-related protein concentrations were greater in MHCC97H-OXA cells compared to parental MHCC97H cells, and also were suppressed by PQ401 treatment.

## Discussion

For patients with advanced HCC, TACE and systemic chemotherapy are the most commom methods of treatment. These therapies often effectively shrink the tumor initially but ultimately fail to eliminate all cancerous tissue, and even leading to tumor relapse. This represents a major challenge in cancer treatment. Additionally, tumor chemoresistance can develop as a result of decreased drug uptake, increased drug efflux, activation of detoxifying systems or DNA repair mechanisms, and/or evasion of drug-induced apoptosis. This is an evidence that tumor chemoresistance is driven by CSCs [35].

Cancer stem cells are the cells within a tumor that possess the capacity to self-renewal and to cause the heterogeneous lineages of cancer cells that comprise the tumor [36]. Most cancer stem cells have been identified by a specific biomarkers and different tissue sources of cancer stem cells have a different biomarkers. For example, CD133, a pentaspan membrane glycoprotein, has been used as a stem cell biomarker for isolation of stem-like cells from a variety of normal and pathological tissues [37]. Some studies showed that CD133+ liver cancer cells are liver cancer stem cell [38], however, others suggested that CD90+ and CD44+ are the biomarkers of liver cancer stem cell [14].It is because of this, we had chosen as much more accepted and several related markers of liver cancer stem cells to confirm the presence of stemness. The behavior of CSCs is critically dependent on several signaling pathways such as the Wnt/β-catenin, Notch, Hedgehog, fibroblast growth factor, transforming growth factor-beta/bone morphogenic protein, and PI3K/AKT/mTOR pathways [39]. Studies have shown that CSC signal transduction pathways are activated by cytokines released by stromal cells such as cancer-associated fibroblasts [40], endothelial cells [41], and a variety of immunological cells including lymphocytes and tumor-associated macrophages [42]. In this study, we explored the cytokines was secreted by tumor cells in the importance of maintaining tumor stemness.

The article "Maintenance of Stemness in Oxaliplatin-Resistant Hepatocellular Carcinoma Is Associated with Increased Autocrine of IGF1" was retracted in 2025. Reasons: errors in the data; errors in the images; duplicated images; overlap with earlier publications.

Although oxaliplatin is widely used in the treatment of advanced malignancies, it is far from being satisfactory for long-term treatment outcome. We had shown that HCC cells still were alive in oxaliplatin treatment (i.e., s.c. tumors from oxaliplatin-treated mice that were orthotopically xenografted into livers of other mice) and underwent EMT, obtained more oxaliplatin-resistant, and demonstrated increasing pulmonary metastatic potential [10]. We also showed that the increased chemoresistance of HCC cells from oxaliplatin-treated mice may be due to enhanced stemness [43]. We used DNA microarrays to compare gene expression profiles of HCC orthotopic xenografts from both oxaliplatin-treated and control mice, and found that the gene for IGF1 was significantly up-regulated. We then established oxaliplatin-resistant HCC cells (MHCC97H-OXA cells) which demonstrated enhancing chemoresistance, invasiveness, cell colony formation, and significantly increasing IGF1 secretion. The IGF1 pathway has been implicated in the etiology of several epithelial malignancies, including liver, breast, colon, prostate, and gynecologic cancers [44]. Sivakumar et al. [45] reported that IGF1R, which is an important receptor tyrosine kinase involved in IGF1-mediated mitogenic signaling, is also critically involved in EMT. Adhami et al. [24] reported the IGF1 axis as a pathway for cancer chemoprevention. Bitelman et al. [46] reported that cisplatin-resistant cells demonstrating increased activation of the IGF1 pathway recovered their sensitivity to cisplatin after small interfering RNA treatment. IGF1R activation has been known to protect tumor cells against apoptosis induced by cytotoxic drugs, and may also influence the repair of DNA damage [47]. From our research and the other results cited here, it is clear that activation of the IGF1 pathway is relevant to the maintenance of stemness.

The article "Maintenance of Stemness in Oxaliplatin-Resistant Hepatocellular Carcinoma Is Associated with Increased Autocrine of IGF1" was retracted in 2025. Reasons: errors in the data; errors in the images; duplicated images; overlap with earlier publications.

Several IGF1R inhibitors have been developed in recent years, some of which have been used in Phase I–III clinical trials as monotherapy as well as in combination with chemo- or radiotherapy. There are considerable preclinical data to support the view that IGF1R inhibition can modify sensitivity to chemical and biological therapies [48], [49]. In the present study, we found that surviving HCC cells in oxaliplatin treatment, which demonstrating enhanced stemness and increased secretion of IGF1. Additionally, the stemness of MHCC97H-OXA cells was inhibited by IGF1R inhibitor PQ401, indicating that the increased autocrine of IGF1 in maintaining stemness had been effectively abolished. Rochester et al. [50] reported that IGF1R knockdown enhancing sensitivity to mitoxantrone, etoposide, nitrogen mustard, and ionizing radiation in human prostate cancer cells. There is other evidence that IGF1R inhibition can prolong the response to endocrine therapy in a murine prostate cancer model [51]. These results suggest that combining oxaliplatin treatment and IGF1R inhibition has potential clinical significance for improving efficiency of oxaliplatin-based chemotherapy regimens.

Intracellular signaling pathways are implicated in cancer cell proliferation and survival and CSC self-renewal depending upon continuous stimulation by extracellular cytokines. Without appropriate stimulation, CSCs will differentiate into common tumor cells. Similarly, EMT tumor cells will undergo mesenchymal-epithelial transition (MET) when cells leave the primary tumor niche [52]. IGF1 plays an important role in the activation of IGF1R signaling, which is related to maintenance of stemness. It is also an autocrine and paracrine factor produced by tumor stromal cells and parenchymal cells. Therefore, IGF1R blocking could effectively interfere with the maintenance of stemness and increase chemotherapeutic sensitivity to oxaliplatin.

## Conclusion

Maintenance of stemness in oxaliplatin-resistant hepatocellular carcinoma is associated with increased autocrine of IGF1.

## References

[1] JemalA, BrayF, CenterMM, FerlayJ, WardE, et al (2011) Global cancer statistics. CA Cancer J Clin 61: 69–90.2129685510.3322/caac.20107

[2] YeSL, TakayamaT, GeschwindJ, MarreroJA, BronowickiJP (2010) Current approaches to the treatment of early hepatocellular carcinoma. Oncologist 15 Suppl 434–41.2111557910.1634/theoncologist.2010-S4-34

[3] BruixJ, SalaM, LlovetJM (2004) Chemoembolization for hepatocellular carcinoma. Gastroenterology 127: S179–188.1550808310.1053/j.gastro.2004.09.032

[4] El-SeragHB (2011) Hepatocellular carcinoma. N Engl J Med 365: 1118–1127.2199212410.1056/NEJMra1001683

The article "Maintenance of Stemness in Oxaliplatin-Resistant Hepatocellular Carcinoma Is Associated with Increased Autocrine of IGF1" was retracted in 2025. Reasons: errors in the data; errors in the images; duplicated images; overlap with earlier publications.

[5] YenY, LimDW, ChungV, MorganRJ, LeongLA, et al (2008) Phase II study of oxaliplatin in patients with unresectable, metastatic, or recurrent hepatocellular cancer: a California Cancer Consortium Trial. Am J Clin Oncol 31: 317–322.1884598810.1097/COC.0b013e318162f57d

[6] YangAD, FanF, CampER, van BurenG, LiuW, et al (2006) Chronic oxaliplatin resistance induces epithelial-to-mesenchymal transition in colorectal cancer cell lines. Clin Cancer Res 12: 4147–4153.1685778510.1158/1078-0432.CCR-06-0038

[7] ShahAN, SummyJM, ZhangJ, ParkSI, ParikhNU, et al (2007) Development and characterization of gemcitabine-resistant pancreatic tumor cells. Ann Surg Oncol 14: 3629–3637.1790991610.1245/s10434-007-9583-5

[8] De LarcoJE, WuertzBR, ManivelJC, FurchtLT (2001) Progression and enhancement of metastatic potential after exposure of tumor cells to chemotherapeutic agents. Cancer Res 61: 2857–2861.11306458

[9] KajiyamaH, ShibataK, TerauchiM, YamashitaM, InoK, et al (2007) Chemoresistance to paclitaxel induces epithelial-mesenchymal transition and enhances metastatic potential for epithelial ovarian carcinoma cells. Int J Oncol 31: 277–283.17611683

[10] XiongW, RenZG, QiuSJ, SunHC, WangL, et al (2010) Residual hepatocellular carcinoma after oxaliplatin treatment has increased metastatic potential in a nude mouse model and is attenuated by Songyou Yin. BMC Cancer 10: 219.2048754210.1186/1471-2407-10-219PMC2880993

[11] YamauchiK, YangM, HayashiK, JiangP, YamamotoN, et al (2008) Induction of cancer metastasis by cyclophosphamide pretreatment of host mice: an opposite effect of chemotherapy. Cancer Res 68: 516–520.1819954710.1158/0008-5472.CAN-07-3063

[12] YamashitaT, JiJ, BudhuA, ForguesM, YangW, et al (2009) EpCAM-positive hepatocellular carcinoma cells are tumor-initiating cells with stem/progenitor cell features. Gastroenterology 136: 1012–1024.1915035010.1053/j.gastro.2008.12.004PMC2828822

[13] LeeTK, CastilhoA, CheungVC, TangKH, MaS, et al (2011) CD24(+) liver tumor-initiating cells drive self-renewal and tumor initiation through STAT3-mediated NANOG regulation. Cell Stem Cell 9: 50–63.2172683310.1016/j.stem.2011.06.005

[14] YangZF, HoDW, NgMN, LauCK, YuWC, et al (2008) Significance of CD90+ cancer stem cells in human liver cancer. Cancer Cell 13: 153–166.1824251510.1016/j.ccr.2008.01.013

[15] LiuLL, FuD, MaY, ShenXZ (2011) The power and the promise of liver cancer stem cell markers. Stem Cells Dev 20: 2023–2030.2165138110.1089/scd.2011.0012

[16] DeanM, FojoT, BatesS (2005) Tumour stem cells and drug resistance. Nat Rev Cancer 5: 275–284.1580315410.1038/nrc1590

[17] JordanCT, GuzmanML (2004) Mechanisms controlling pathogenesis and survival of leukemic stem cells. Oncogene 23: 7178–7187.1537807810.1038/sj.onc.1207935

The article "Maintenance of Stemness in Oxaliplatin-Resistant Hepatocellular Carcinoma Is Associated with Increased Autocrine of IGF1" was retracted in 2025. Reasons: errors in the data; errors in the images; duplicated images; overlap with earlier publications.

[18] CostelloRT, MalletF, GauglerB, SaintyD, ArnouletC, et al (2000) Human acute myeloid leukemia CD34+/CD38- progenitor cells have decreased sensitivity to chemotherapy and Fas-induced apoptosis, reduced immunogenicity, and impaired dendritic cell transformation capacities. Cancer Res 60: 4403–4411.10969785

[19] LiuG, YuanX, ZengZ, TuniciP, NgH, et al (2006) Analysis of gene expression and chemoresistance of CD133+ cancer stem cells in glioblastoma. Mol Cancer 5: 67.1714045510.1186/1476-4598-5-67PMC1697823

[20] BodzinAS, WeiZ, HurttR, GuT, DoriaC (2012) Gefitinib resistance in HCC mahlavu cells: upregulation of CD133 expression, activation of IGF-1R signaling pathway, and enhancement of IGF-1R nuclear translocation. J Cell Physiol 227: 2947–2952.2195979510.1002/jcp.23041

[21] FordNA, NunezNP, HolcombVB, HurstingSD (2013) IGF1 dependence of dietary energy balance effects on murine Met1 mammary tumor progression, epithelial-to-mesenchymal transition, and chemokine expression. Endocr Relat Cancer 20: 39–51.2315244210.1530/ERC-12-0329

[22] PngKJ, HalbergN, YoshidaM, TavazoieSF (2012) A microRNA regulon that mediates endothelial recruitment and metastasis by cancer cells. Nature 481: 190–194.10.1038/nature1066122170610

[23] ChitnisMM, YuenJS, ProtheroeAS, PollakM, MacaulayVM (2008) The type 1 insulin-like growth factor receptor pathway. Clin Cancer Res 14: 6364–6370.1892727410.1158/1078-0432.CCR-07-4879

[24] AdhamiVM, AfaqF, MukhtarH (2006) Insulin-like growth factor-I axis as a pathway for cancer chemoprevention. Clin Cancer Res 12: 5611–5614.1702096210.1158/1078-0432.CCR-06-1564

[25] PollakM (2008) Insulin, insulin-like growth factors and neoplasia. Best Pract Res Clin Endocrinol Metab 22: 625–638.1897112310.1016/j.beem.2008.08.004

[26] LeeJ, JuJ, ParkS, HongSJ, YoonS (2012) Inhibition of IGF-1 signaling by genistein: modulation of E-cadherin expression and downregulation of beta-catenin signaling in hormone refractory PC-3 prostate cancer cells. Nutr Cancer 64: 153–162.2209810810.1080/01635581.2012.630161

[27] LeeTK, CastilhoA, CheungVC, TangKH, MaS, et al (2011) Lupeol targets liver tumor-initiating cells through phosphatase and tensin homolog modulation. Hepatology 53: 160–170.2097905710.1002/hep.24000

[28] SunayamaJ, MatsudaK, SatoA, TachibanaK, SuzukiK, et al (2010) Crosstalk between the PI3K/mTOR and MEK/ERK pathways involved in the maintenance of self-renewal and tumorigenicity of glioblastoma stem-like cells. Stem Cells 28: 1930–1939.2085749710.1002/stem.521

[29] WangYK, ZhuYL, QiuFM, ZhangT, ChenZG, et al (2010) Activation of Akt and MAPK pathways enhances the tumorigenicity of CD133+ primary colon cancer cells. Carcinogenesis 31: 1376–1380.2053055410.1093/carcin/bgq120

The article "Maintenance of Stemness in Oxaliplatin-Resistant Hepatocellular Carcinoma Is Associated with Increased Autocrine of IGF1" was retracted in 2025. Reasons: errors in the data; errors in the images; duplicated images; overlap with earlier publications.

[30] TianJ, TangZY, YeSL, LiuYK, LinZY, et al (1999) New human hepatocellular carcinoma (HCC) cell line with highly metastatic potential (MHCC97) and its expressions of the factors associated with metastasis. Br J Cancer 81: 814–821.1055575110.1038/sj.bjc.6690769PMC2374300

[31] YeQH, QinLX, ForguesM, HeP, KimJW, et al (2003) Predicting hepatitis B virus-positive metastatic hepatocellular carcinomas using gene expression profiling and supervised machine learning. Nat Med 9: 416–423.1264044710.1038/nm843

[32] ZhangT, SunHC, XuY, ZhangKZ, WangL, et al (2005) Overexpression of platelet-derived growth factor receptor alpha in endothelial cells of hepatocellular carcinoma associated with high metastatic potential. Clin Cancer Res 11: 8557–8563.1636153710.1158/1078-0432.CCR-05-0944

[33] MacfarlanTS, GiffordWD, DriscollS, LettieriK, RoweHM, et al (2012) Embryonic stem cell potency fluctuates with endogenous retrovirus activity. Nature 487: 57–63.2272285810.1038/nature11244PMC3395470

[34] XiaoY, IsaacsSN (2012) Enzyme-linked immunosorbent assay (ELISA) and blocking with bovine serum albumin (BSA)–not all BSAs are alike. J Immunol Methods 384: 148–151.2273219410.1016/j.jim.2012.06.009PMC3432671

[35] AlisonMR, LimSM, NicholsonLJ (2011) Cancer stem cells: problems for therapy? J Pathol 223: 147–161.2112567210.1002/path.2793

[36] ClarkeMF, DickJE, DirksPB, EavesCJ, JamiesonCH, et al (2006) Cancer stem cells–perspectives on current status and future directions: AACR Workshop on cancer stem cells. Cancer Res 66: 9339–9344.1699034610.1158/0008-5472.CAN-06-3126

[37] LiZ (2013) CD133: a stem cell biomarker and beyond. Exp Hematol Oncol 2: 17.2381581410.1186/2162-3619-2-17PMC3701589

[38] MaS, LeeTK, ZhengBJ, ChanKW, GuanXY (2008) CD133+ HCC cancer stem cells confer chemoresistance by preferential expression of the Akt/PKB survival pathway. Oncogene 27: 1749–1758.1789117410.1038/sj.onc.1210811

[39] TongCM, MaS, GuanXY (2011) Biology of hepatic cancer stem cells. J Gastroenterol Hepatol 26: 1229–1237.2155777010.1111/j.1440-1746.2011.06762.x

[40] GiannoniE, BianchiniF, MasieriL, SerniS, TorreE, et al (2010) Reciprocal activation of prostate cancer cells and cancer-associated fibroblasts stimulates epithelial-mesenchymal transition and cancer stemness. Cancer Res 70: 6945–6956.2069936910.1158/0008-5472.CAN-10-0785

[41] LuJ, YeX, FanF, XiaL, BhattacharyaR, et al (2013) Endothelial cells promote the colorectal cancer stem cell phenotype through a soluble form of Jagged-1. Cancer Cell 23: 171–185.2337563610.1016/j.ccr.2012.12.021PMC3574187

The article "Maintenance of Stemness in Oxaliplatin-Resistant Hepatocellular Carcinoma Is Associated with Increased Autocrine of IGF1" was retracted in 2025. Reasons: errors in the data; errors in the images; duplicated images; overlap with earlier publications.

[42] SicaA, LarghiP, MancinoA, RubinoL, PortaC, et al (2008) Macrophage polarization in tumour progression. Semin Cancer Biol 18: 349–355.1846712210.1016/j.semcancer.2008.03.004

[43] JiaQA, RenZG, BuY, WangZM, ZhangQB, et al (2012) Herbal Compound “Songyou Yin” Renders Hepatocellular Carcinoma Sensitive to Oxaliplatin through Inhibition of Stemness. Evid Based Complement Alternat Med 2012: 908601.2332629310.1155/2012/908601PMC3541605

[44] WernerH, BruchimI (2009) The insulin-like growth factor-I receptor as an oncogene. Arch Physiol Biochem 115: 58–71.1948570210.1080/13813450902783106

[45] SivakumarR, KogaH, SelvendiranK, MaeyamaM, UenoT, et al (2009) Autocrine loop for IGF-I receptor signaling in SLUG-mediated epithelial-mesenchymal transition. Int J Oncol 34: 329–338.19148466

[46] Bitelman C, Sarfstein R, Sarig M, Attias-Geva Z, Fishman A, et al. (2013) IGF1R-directed targeted therapy enhances the cytotoxic effect of chemotherapy in endometrial cancer. Cancer Lett.10.1016/j.canlet.2013.02.00923402816

[47] SunY, ZhengS, TorossianA, SpeirsCK, SchleicherS, et al (2012) Role of insulin-like growth factor-1 signaling pathway in cisplatin-resistant lung cancer cells. Int J Radiat Oncol Biol Phys 82: e563–572.2219723010.1016/j.ijrobp.2011.06.1999PMC3271860

[48] YuenJS, MacaulayVM (2008) Targeting the type 1 insulin-like growth factor receptor as a treatment for cancer. Expert Opin Ther Targets 12: 589–603.1841024210.1517/14728222.12.5.589

[49] SamaniAA, YakarS, LeRoithD, BrodtP (2007) The role of the IGF system in cancer growth and metastasis: overview and recent insights. Endocr Rev 28: 20–47.1693176710.1210/er.2006-0001

[50] RochesterMA, RiedemannJ, HellawellGO, BrewsterSF, MacaulayVM (2005) Silencing of the IGF1R gene enhances sensitivity to DNA-damaging agents in both PTEN wild-type and mutant human prostate cancer. Cancer Gene Ther 12: 90–100.1549937810.1038/sj.cgt.7700775

[51] PlymateSR, HaugkK, ColemanI, WoodkeL, VessellaR, et al (2007) An antibody targeting the type I insulin-like growth factor receptor enhances the castration-induced response in androgen-dependent prostate cancer. Clin Cancer Res 13: 6429–6439.1797515510.1158/1078-0432.CCR-07-0648

[52] BrabletzT (2012) EMT and MET in metastasis: where are the cancer stem cells? Cancer Cell 22: 699–701.2323800810.1016/j.ccr.2012.11.009

